RETRACTED

# Clinical Study of Anti-PD-1 Immunotherapy Combined with Gemcitabine Chemotherapy in Multiline Treatment of Advanced Pancreatic Cancer

**DOI:** 10.1155/2022/4070060

**Published:** 2022-09-06

**Authors:** Yanfeng Liu, Yanchuan Li, Shan Du, Li Fan, Junyan Wang

**Affiliations:** ^1^General Surgery Department, The Second Affiliated Hospital of Xi'an Medical University, Xi'an, Shaanxi 710038, China; ^2^Gynaecology and Obstetrics Department, Shaanxi Provincial People's Hospital, Xi'an, Shaanxi 710068, China; ^3^Gastroenterology Department, The Second Affiliated Hospital of Xi'an Medical University, Xi'an, Shaanxi 710038, China

## Abstract

**Objective:**

This study aimed to investigate the efficacy and safety of anti-PD-1 immunotherapy combined with gemcitabine chemotherapy in multiline treatment of advanced pancreatic cancer.

**Methods:**

A retrospective analysis was performed on the clinical data of 32 patients with advanced pancreatic cancer treated with sintilimab regimen from January 2019 to December 2021 in our hospital. All patients were followed up until death or April 2022, in the form of outpatient, in-hospital review, or telephone follow-up. Follow-up content included routine blood, liver and kidney functions, tumor markers, plain or enhanced abdominal CT, and abdominal MRI examinations. Clinical efficacy was evaluated according to mRECIST criteria, and the severity of adverse effects was evaluated according to American Institute for Cancer Research (AICR) Standard Term for Adverse Events, Version 5.0.

**Results:**

During treatment, the dosage of sintilimab was halved in 2 patients due to adverse reactions. All patients were treated with sintilimab for 1~10 times, with an average of 6 ± 4 times. The total response rate (ORR) and disease control rate (DCR) were 6.25% and 12.50% and 25.00% and 37.50%, respectively, after 1 and 3 months of treatment. The mean follow-up time of 32 patients was 1-12 months, and the median follow-up time was 4 ± 3 months. By the end point of follow-up, a total of 25 patients died, and the median progression-free survival (PFS) was 3.8 (95% CI (1.85-5.63)) months. The median overall survival (OS) was 5.1 months (95% CI (3.63~7.68). After treatment, the levels of tumor markers CA125, CEA and CA199 were partly decreased compared with those before treatment (all *P* < 0.001). After treatment, the blood routine indexes d-dimer, CRP (C-reactive protein), NLR (neutral granulocyte to lymphocyte ratio), and MLR (monocyte to lymphocyte ratio) decreased compared with those before treatment. In 32 patients with advanced pancreatic cancer, the adverse reactions with an incidence more than 10% included fatigue, rash, hypothyroidism, hyperuricemia, and renal insufficiency. Only 2 patients showed grade 3 fatigue symptom, and all the others showed no adverse reactions of grades 3~5. In this study, all patients' adverse reactions were relieved after symptomatic treatment.

RETRACTED

**Conclusion:**

Gemcitabine chemotherapy in multiline treatment of advanced pancreatic cancer with sintilimab can achieve certain clinical benefits without serious adverse reactions.

## 1. Introduction

Pancreatic cancer is one of the malignant tumors of the digestive system with the highest mortality, accounting for the fourth place in the cancer-related mortality [1, 2]. In recent years, epidemiology has found that the number of new pancreatic cancer cases in both male and female is increasing [3, 4]. In the USA, the number of new malignant tumors ranks 10th in men and 9th in women among all tumors [5], and in China, the number ranks 7th in men and 11th in women [6]. The annual incidence of pancreatic cancer is 12.9 cases/100,000 person-years. However, pancreatic cancer has a poor prognosis, with a mortality rate of 11 cases/100,000 person-years [7]. Most patients are found in the middle and late stages and lose the opportunity for surgical treatment. Standardized, reasonable, and scientific drug treatment can prolong the survival of patients with middle and advanced pancreatic cancer [8]. With the deepening of imaging, endoscopic technology and pathological research, and the continuous development of surgical treatment technology and local treatment technology, the treatment status of patients with pancreatic cancer has been significantly improved, and the number of patients with long-term survival has also been increasing [9, 10]. At present, the effective treatment of pancreatic cancer is still based on surgery, supplemented by radiation therapy and chemotherapy. With the deepening of research on tumorigenesis, development and metastasis mechanism of immune and molecular biology, gene therapy, and immunotherapy of pancreatic cancer become possible, and they also becomes new development direction of pancreatic cancer treatment [11]. Programmed death receptor-1 (PD-1) is a transmembrane protein belonging to the B7H3 immune superfamily. It is widely expressed in activated T lymphocytes, monocytes, B cells, natural killer cells, and dendritic cells and participates in immune surveillance and maintenance of immune tolerance [12, 13]. PD-1 and its ligand are also highly expressed in pancreatic cancer tumor cells [14]. Immunotherapy with PD-1 inhibitor as the main treatment scheme has achieved definite efficacy in a variety of solid tumor patients [15, 16]. Sintilimab (trade name: Daboshu) is a fully humanized IgG4 monoclonal antibody targeting PD-1. In 2018, it was approved by China's State Drug Administration (SDA) for clinical treatment of malignant tumors, and several phase I and phase II clinical trials were conducted at the same time [17–19]. At present, there are relatively few domestic clinical reports on the treatment of advanced pancreatic cancer with sintilimab combined with traditional chemotherapy drugs. This study conducted a retrospective analysis on the treatment of advanced pancreatic cancer with sintilimab in our hospital. The results are reported as follows.

RETRACTED

## 2. Subjects and Methods

### 2.1. Research Subjects

The clinical data of patients with pancreatic cancer admitted to our hospital from January 2019 to December 2021 were retrospectively analyzed. All patients signed the informed consent form, and the study design was in line with the Declaration of Helsinki. Inclusion criteria are as follows: (1) Patients met the diagnostic criteria for pancreatic cancer in the Guidelines for Comprehensive Diagnosis and Treatment of Pancreatic Cancer in China (2020 version) [20]; (2) patients with locally advanced inoperable, metastatic, and postoperative recurrence and metastasis of pancreatic cancer; (3) the pathological type was adenocarcinoma; (4) the survival time can be followed up; (5) gemcitabine was included in the chemotherapy regimen; and (6) complete clinical data. Exclusion criteria are as follows: (1) The estimated survival was less than 3 months; (2) the tumor stage was stage IV; (3) patients had no indication of surgery or radiotherapy or who give up treatment; (4) patients had symptomatic brain metastases; (5) patients who have received chemotherapy in the past; and (6) immunodeficiency patients. A total of 32 patients with sintilimab included in the treatment regimen were selected. All patients had not received radiotherapy and chemotherapy before enrollment.

### 2.2. Therapies

Sintilimab Injection (Innovent; SFDA approval number: S20180016) was administrated once every 3 weeks with a dose of 200 mg. Gemcitabine hydrochloride for injection (produced by Jiangsu Hausen Pharmaceutical Group, National drug Approval H20030104) was dissolved in 100 mL normal saline at 1000 g/m^2^ and given intravenously for 30 min on the 1st and 8th days. Both were used until disease progression, severe adverse reactions, or self-termination of treatment.

### 2.3. Follow-Up and Outcome Evaluation

All patients were followed up until death or April 2022, in the form of outpatient, in-hospital review, or telephone follow-up. Follow-up content included routine blood, liver and kidney functions, tumor markers, plain or enhanced abdominal CT, and abdominal MRI examinations.

RETRACTED

Efficacy evaluation: Clinical efficacy was evaluated according to mRECIST criteria [21]. The efficacy of CT or MRI reexamination results of patients at 1 and 3 months of treatment were divided into complete response (CR), partial response (PR), stable disease (SD), and progressive disease (PD), and the total response rate (ORR) and disease control rate (DCR) were calculated according to ORR = CR + PR and DCR = CR + PR + SD.

Adverse reactions: The severity of toxic side effects in patients enrolled in this study was evaluated according to American Institute for Cancer Research (AICR) Standard Term for Adverse Events, Version 5.0 [22]. The toxic side effects were divided into levels 1 to 5, and the higher the level, the more serious the adverse effects were. The evaluation time was within 28 days after the last administration. The toxic side effects of included events include fatigue, skin rash, hypothyroidism, hyperuricemia, and renal insufficiency.

Two fixed physicians with extensive clinical experience evaluated efficacy and adverse effects. If there was any objection, please ask the third physician to further discuss and clarify.

### 2.4. Statistical Analysis

SPSS23.0 was used to analyze the collected experimental data. Mean ± standard deviation (*X* ± *S*) was used to represent the measurement data in accordance with normal distribution, and the counting data was expressed as cases or rates. Kaplan-Meier method was used to plot survival curves and count the progression-free survival (PFS) and overall survival (OS).

## 3. Results

### 3.1. Baseline Data

The baseline data of enrolled patients are shown in Table 1.

### 3.2. Short-Term Efficacy Evaluation

By the end of follow-up, the effective follow-up information of all 32 patients was obtained, and no one withdrew from the study due to serious adverse reactions or other reasons. During treatment, the dosage of sintilimab was halved in 2 patients due to adverse reactions. All patients were treated with sintilimab for 1~10 times, with an average of 6 ± 4 times. The ORRs at 1 and 3 months after treatment are 6.25% and 12.50%, respectively, and the DCRs are 25.00% and 37.50%, respectively, as shown in Table 2.

### 3.3. Survival Benefit Evaluation

The mean follow-up time of the 32 patients was 1-12 months, and the median follow-up time was 4 ± 3 months. By the end point of follow-up, a total of 25 patients died, with a median PFS of 3.8 (95% CI (1.85-5.63)) months and a median OS of 5.1 months (95% CI (3.63-7.68)), as shown in Figure 1.

### 3.4. Evaluation of Tumor Markers before and after Treatment

After treatment, the levels of tumor markers CA125, CEA, and CA199 are partly decreased compared with those before treatment (all *P* < 0.001), as shown in Table 3.

RETRACTED

### 3.5. Evaluation of Blood Routine Indexes before and after Treatment

After treatment, the blood routine indexes D-dimer, CRP, NLR, and MLR all significantly decrease compared with those before treatment (all *P* < 0.05), as shown in Table 4.

### 3.6. Evaluation of Adverse Reactions

According to the AICR Standard Term for Adverse Events version 5.0, the adverse reactions with an incidence more than 10% in these 32 patients included fatigue, rash, hypothyroidism, hyperuricemia, and renal insufficiency. Only 2 patients showed grade 3 fatigue symptom, and all the others showed no adverse reactions of grades 3~5. All patients in this study are relieved after symptomatic treatment, as shown in Table 5.

## 4. Discussion

Epidemiological investigation found that the absolute and relative numbers of incidence and death of pancreatic cancer in China increased significantly in 2019 compared with 1990, with the normalized incidence and mortality increasing by 82.33% and 79.34%, indicating that the burden of pancreatic cancer on the health of Chinese residents is gradually increasing [23, 24]. In terms of morbidity characteristics, male, age, diet, and alcohol have significant influence on the incidence of pancreatic cancer in Chinese residents [25]. As a highly invasive malignant tumor with high mortality, about 60% of them have metastasis at first diagnosis, about 30% have been in local progression at first diagnosis, and only 15% can receive radical surgery. Most patients die due to tumor metastasis or recurrence, with the 5-year survival rate being only 7% [26]. Anti-PD-1 monoclonal antibody has been approved for a short time in China, but its therapeutic effect in a variety of solid tumors has been confirmed. The present study analyzed the efficacy and safety of the multiline treatment regimen containing sintilimab in patients with advanced pancreatic cancer, with the aim of enriching the clinical data and providing a valuable reference for the promotion and application of this drug.

Studies [27, 28] found that therapies combined with immune checkpoints can regulate the immune editing process of pancreatic cancer tissues and directly affect the tumor microenvironment and immune response behavior. Drug combination can also overcome the resistance of pancreatic cancer to PD-1/PD-L1 monotherapy and promote the transformation of tumor biological behavior from nonimmunological to immunological, which maximizes the antitumor therapeutic effects of immunosuppressants [29]. The combination of PD-L1 blocker and gemcitabine has been proved to have antitumor effect in the treatment of pancreatic cancer, while the clinical response rate of the combination of pembrolizumab/gemcitabine + albumin-bound paclitaxel in the treatment of pancreatic cancer is up to 92% [29]. An in vitro study [30] found that sintilimab can specifically bind human PD-1 in high concentration and block the binding of PD-1 with PD-L1/PD-l2 ligand. When the dose of sintilimab injection is 200 mg, it can rapidly occupy more than 95% of PD-1 receptors on the surface of T cells. In addition, sintilimab can significantly increase the levels of interleukin-2 and interferon-ƴ in a dose-dependent manner, which may be one of the molecular mechanisms for its antitumor role [31].

RETRACTED

This study analyzed the clinical data of 32 patients with advanced pancreatic cancer who received sintilimab multiline therapy in our hospital. The results showed that the dosage of sintilimab was halved in 2 patients due to adverse reactions during the treatment. The ORR of 1 month and 3 months after treatment was 6.25% and 12.50%, respectively, and the DCR was 25.00% and 37.50%, respectively. In the study of Xiao Xia et al. [32], among 8 patients with advanced pancreatic cancer treated with sintilimab, 1 patient had PR, 1 patient had SD, and 6 patients had PD. Objective remission was observed in 1 case and disease control in 2 cases. The median PFS was 2.0 months (95% CI 0.6-3.4 months), and the median OS was 3.5 months (95% CI 2.2-4.8 months), which were similar to the results of our study. However, in the study of Le et al. [33], the disease control rate in dMMR or MSI-H-positive patients with advanced metastatic pancreatic cancer treated with anti-PD-1 monoclonal antibody is up to 75%. In addition, it was reported that the disease control rate of patients with metastatic pancreatic cancer treated with pembrolizumab combined with chemotherapy is up to 100% [34]. The reasons for the differences among different studies may be related to drug dosage, heterogeneity of patients' baseline data, and differences in sample size. In the present study, the mean follow-up time of 32 patients was 1-12 months, and the median follow-up time was 4 ± 3 months. By the end point of follow-up, a total of 25 patients died, with a median PFS of 3.8 (95% CI (1.85-5.63)) months and a median OS of 5.1 months (95% CI (3.63-7.68)). Compared with the results of Xiao Xia et al., both PFS and OS in our study were improved to a certain extent, suggesting that sintilimab combined with chemotherapy had certain clinical benefits in the multiline treatment of advanced pancreatic cancer.

In terms of efficacy evaluation indexes, the levels of tumor markers CA125, CEA, and CA199 decreased significantly after treatment compared with before treatment, and the blood routine indexes (D-dimer, CRP, NLR, and MLR) decreased after treatment compared with before treatment, indicating that hematological indexes had certain value in evaluating the efficacy of this treatment regimen. However, whether its application value is better than that of serum PD-1 and PD-L1 as well as the optimal threshold of single indicator and multiple indicator combination needs further discussion.

RETRACTED

It has been reported [35] that while promoting tumor immune response, sintilimab may lead to excessive immune response, induce autoimmune response, and cause immune-related adverse events in skin, gastrointestinal tract, liver, kidney, and endocrine system. The results of our study showed that the adverse reactions with an incidence over 10% during treatment included fatigue, rash, hypothyroidism, hyperuricemia, and renal insufficiency. Only 2 patients had grade 3 fatigue symptoms, and the rest had no grades 3-5 adverse reactions. In this study, all patients' adverse reactions were alleviated after symptomatic treatment, indicating that this treatment plan did not cause serious treatment-related adverse reactions and was safe.

Overall, the results of this study suggested that patients with advanced pancreatic cancer can benefit from the multiline therapy with sintilimab, with no serious adverse reactions. However, according to other studies, there are still many problems with anti-PD-1 monoclonal antibody drugs in the treatment of pancreatic cancer. For example, about half of patients have poor response efficiency to pD-1/PD-L1 treatment but lack relevant evaluation markers. Anti-PD-1/PD-L1 monotherapy for solid tumors has poor efficacy and is mostly used in combination, and the optimal combination plan still needs to be discussed. In addition, the high cost of anti-PD-1/PD-L1 treatment restricts its promotion [36], which is one of the reasons for the small sample size reported in most cases. And this study lacked a noncombination control group. Interleukin-2 and interferon-ƴ can be detected to evaluate the antitumor effect. Future follow-up studies need to expand the sample size and follow-up time to develop the best treatment plan to maximize the clinical benefit of patients. And future follow-up studies will improve the control group settings and detect immune indicators to evaluate the antitumor effect.

## Figures and Tables

**Figure 1:** Survival curve of sintilimab immunotherapy regimen.

**Table 1:** Comparison of baseline data between two groups.

Item		Sintilimab (*n* = 32)
Gender	Male	19
	Female	13
Age (years)		58.37 ± 10.53
Body mass index (kg/m^2^)		22.18 ± 2.53
Complicated with diabetes		6
Complicated with hypertension		7
Tumor site	Uncinate process of pancreatic head	20
	Body and tail of pancreas	12
Nerve infiltration	Yes	14
	No	18
Degree of differentiation	Low/medium differentiation	19
	Highly differentiation	13

RETRACTED

**Table 2:** Short-term efficacy evaluation.

Time point	CR	PR	SD	PD	ORR	DCR
1 month	0 (0)	2 (6.25)	6 (18.75)	24 (75.00)	2 (6.25)	8 (25.00)
3 months	0 (0)	4 (12.50)	8 (25.00)	20 (62.50)	4 (12.5)	12 (37.50)

Note: CR: complete remission; PR: partial remission; SD: stable disease; PD: progressive disease; ORR: overall response rate.

**Table 3:** Evaluation of tumor markers before and after treatment.

Index	Before treatment	After treatment	*P* value
CA125	10.53 ± 7.34	7.83 ± 5.83	<0.001
CEA	464.53 ± 386.74	416.34 ± 32.53	<0.001
CA199	49.37 ± 40.83	40.86 ± 38.76	<0.001

**Table 4:** Evaluation of blood routine indexes before and after treatment.

Index	Before treatment	After treatment	*P* value
D-dimer	30.34 ± 13.23	22.38 ± 12.86	<0.001
CRP	28.53 ± 12.76	20.67 ± 12.78	<0.001
NLR	3.43 ± 1.86	2.80 ± 1.79	<0.001
MLR	2.86 ± 1.39	2.28 ± 1.28	<0.001

**Table 5:** Evaluation of adverse reactions (*n*, %).

Adverse reactions	Total incidence	Incidence of grades 3-5 adverse reactions
Fatigue	20 (62.50)	2 (6.25)
Rash	10 (31.25)	0 (0.00)
Hypothyroidism	8 (25.00)	0 (0.00)
Hyperuricemia	6 (18.75)	0 (0.00)
Renal insufficiency	5 (15.63)	0 (0.00)

## Data Availability

The labeled dataset used to support the findings of this study are available from the corresponding author upon request.
